# Up-regulated *miR-500a* enhances hepatocarcinoma metastasis by repressing PTEN expression

This article has been retracted.

**DOI:** 10.1042/BSR20170837

**Published:** 2017-12-15

**Authors:** Yufeng Zhao, Yuehui Wang, Yaqiang Wang

**Affiliations:** 1 Department of Laboratory Medicine, Huaihe Hospital of Henan University, Kaifeng 475000, Henan, China; 2 Department of Cardiology, Huaihe Hospital of Henan University, Kaifeng 475000, Henan, China

**Keywords:** AKT, Hepatocarcinoma, MiR-500a, Metastasis, PTEN

## Abstract

It has been shown that *miR-500a* may play an important role in the metastasis of hepatocarcinoma. The present study is to explore the influence of *miR-500a* on hepatocarcinoma proliferation and metastasis, and the related molecular mechanism. The levels of *miR-500a* in the serum and tissues of patients with metastatic or non-metastatic hepatocarcinoma or normal people were determined by quantitative reverse transcription-PCR (qRT-PCR). The proliferation, invasion, and cloning of hepatocarcinoma cell lines SMMC-7721 after transfection with mimic *miR-500a* or inhibitor *miR-500a* were determined. Luciferase reported assay was used to explore the relationship between *miR-500a* and phosphatase and tensin homologue (PTEN). Then, the protein expression of PTEN, p-Akt (S473), p-Akt (T308), Akt, p-mTOR, mTOR, p-4E-BP1, 4E-BP1, p-S6K, and S6K in SMMC-7721 cells were also determined by Western blotting. The expression of *miR-500a* in patients with metastatic hepatocarcinoma was significantly higher than the non-metastatic hepatocarcinoma. Overexpression of *miR-500a* promoted the proliferation, invasion, and cloning of SMMC-7721 cells. Luciferase reported assay showed *miR-500a* could directly target at 3′-UTR of PTEN. Overexpression of *miR-500a* significantly reduced the expression of PTEN, and enhanced phosphorylation of Akt, mTOR, S6K, and 4E-BP1. In conclusion, the expression of *miR-500a* was related to the proliferation and metastasis of hepatocarcinoma, which may be partly because of the activation of AKT/mTOR pathway through targetting PTEN.

## Introduction

Hepatocarcinoma is a common and aggressive cancer that is strongly associated with chronic infection by the hepatitis B virus (HBV) [1]. Poor prognosis and patient survival with hepatocarcinoma are largely due to invasion/metastasis and postsurgical recurrence [2]. Invasion and metastasis are fundamental properties of hepatocellular carcinoma (HCC), which has a very high mortality rate. Metastasis is a complex cascade, however, and the underlying molecular mechanisms are far from being fully understood [3].

MiRNAs are a class of endogenous phylogenetically conserved small RNAs (~22 nts) responsible for the post-transcriptional regulation of mRNA translation and stability. They are involved in several biological processes, such as development, apoptosis, proliferation, and differentiation. Aberrant expression of numerous miRNAs has been associated with cancer development [4], and deregulated miRNAs have been linked to molecular pathways involved in neoplastic transformation [5]. Altered expression of miRNAs and the identification of their molecular target genes in hepatocarcinoma have previously been described by our and other groups [6,7]. Therefore, taking advantage of promising *in vivo* studies on miRNAs, this class of molecules may represent a new kind of unconventional targetted treatment to be eventually associated with traditional approaches for hepatocarcinoma not amenable of curative therapies [8]. As previous study showed *miR-500a* was found as an oncofetal miRNA in liver cancer. The increased amount of *miR-500a* was found in the sera of the HCC patients [9]. But the detailed mechanism of *miR-500a* regulating liver cancer is unknown.

The aim of the present study was to investigate the relationship between miRNAs and the proliferation and metastasis of hepatocarcinoma and the related molecular mechanism. First, we determined the level of *miR-500a* in serum and tissues from metastatic and non-metastatic hepatocarcinoma patients. Then, hepatocarcinoma cells were transfected with mimic *miR-500a* or inhibitor *miR-500*a, and the proliferation capacity and invasion of cells were determined. Moreover, we found that *miR-500a* influenced AKT signaling pathway by targetting PTEN.

## Materials and methods

### Serum and tissue samples

Serum samples were obtained from 12 patients with hepatocarcinoma and 17 cases of the normal people to study and compare the expression of *miR-500a*. Moreover, serum and tissues were also obtained from ten cases of non-metastatic hepatocarcinoma patients and seven cases of metastatic hepatocarcinoma patients. All patients underwent surgery in the Huaihe Hospital of Henan University (Henan, China) during February 2013 to November 2015. Before surgery, there had not underwent chemotherapy or radiotherapy.

Peripheral blood was obtained in the early morning from all individuals. Sera were separated by centrifuging the blood samples at 3000 rpm for 15 min. The samples were stored at –80°C or fixed in formaldehyde after resection. All patients’ samples were obtained at their first visit. Clinical and laboratory data reported in the present study were obtained at the time of sampling. The present study was approved by Ethics Committee of Huaihe Hospital of Henan University and written informed consents were obtained before the patients and healthy volunteers entered into the present study.

### RNA isolation

Total RNA was isolated from fresh hepatocarcinoma tissue and serum samples using the miRNeasy Mini Kit (Qiagen, Valencia, CA, U.S.A.) and miRVana RNA isolation kit (Ambion Inc, Austin, TX, U.S.A.) according to the manufacturer’s protocol. RNA purity and concentrations were measured with the Nanodrop 2000 (Thermo Fisher Scientific, San Jose, CA, U.S.A.). RNA integrity was detected on an agarose gel with Ethidium Bromide staining by electrophoresis. The RNA samples were immediately stored at −80°C for next cDNA conversion.

### Cell culture

Human hepatocarcinoma cell lines SMMC-7721 were purchased from the Cell Bank of the Chinese Academy of Sciences (Shanghai, China). The cells were kept in RPMI-1640 medium (Gibco, U.S.A) in humidified air containing 5% CO_2_ at 37°C. RPMI-1640 medium contained 10% FBS (HyClone, U.S.A.) and 1% penicillin/streptomycin.

### Cell transfection

Cells were seeded in six-well plate and cultured overnight. *MiR-500a* mimics, corresponding negative control (mimic NC), the siRNAs targetting *miR-500a* (inhibitor *miR-500a*) and corresponding negative control (inhibitor NC) were synthesized and purified by GenePharma (Shanghai, China). *MiR-500a*-overexpressed plasmid (pCDNA3.1-*miR-500a*) and blank vector pCDNA3.1 were purchased from Chinese Academy of Sciences (Changchun, China). Cells were transfected with the oligonucleotide using Lipofectamine 2000 (Invitrogen, Carlsbad, CA, U.S.A.) according to the manufacturer’s instructions.

### qRT-PCR

Total mRNA was extracted from the retinal samples with TRIzol reagent (Life Technologies, Grand Island, NY) according to the manufacturer’s protocol. Pipette was used to beat upon retinal samples evenly and samples were put into 1.5-ml Eppendorf tubes to stand for 5 min to separate nucleic acid–protein complex. Each EP tube was added with 1 ml TRIzol and 200 μl precooled chloroform. The tubes were shook for 15 s and centrifuged at 4°C, 12000 rpm for 15 min. We drew aqueous phase from other 1.5-ml EP tubes and added 0.5-ml isopropanol. The mixture was mixed and centrifuged at 4°C, 12000 rpm for 15 min. After removing the supernatant, 1 ml precooled 75% ethanol was added to wash RNA precipitate and this procedure was repeated for three times. Then, the RNA precipitate was dried in vacuum and concentration was determined with a NanoDrop 1000 spectrophotometer (NanoDrop Technologies, Wilmington, Delaware, U.S.A.). PCR tubes were prepared, 1 μl oligo dT (0.5 μg/μl) and 2 μg total RNA were put into each tube. After that, diethypyrocarbonate (DEPC) was added into each PCR tube to volume of 12 μl. After mixing evenly, tubes were placed in 65°C water-bath kettle for 5 min and then placed on ice immediately. Reverse transcription was performed at 55°C for 30 min, initial activation for 15 min at 95°C, next 40 cycles of denaturation were conducted at 94°C for 15 s, then annealed for 30 s at 55°C, extension for 30 s at 72°C. The expression level was normalized using U6 snRNA by the 2^−Δ*C*^_t_ method. The Δ*C*_t_ values were normalized to U6 level. Precursor miRNA (pre-miRNA) or the mature miRNA were used as a template for qRT-PCR. The sequence of U6 was RT of AACGCTTCACGAATTTGCGT, F of CTCGCTTCGGCAGCACA and R of AACGCTTCACGA ATTTGCGT. The sequence of *miR-500* was RT of GTCGTATCCAGTGCAGGGTCCG AGGTATTCGCACTGGATACGACTCTCAC, F of TATAA TCCTTGCTACCTGG and R of GTGCAGGGTCCGAGGT. The sequence of cel-*miR-39-3p* was RT of GTCGTATCCAGTGCAGG GTCCGAGGTATTCGCACTGGATACGACCAAGCT, F of TTATCACCGGGTGTAAATC and R of GTGCAGGGTCCGAGGT.

### Western blotting

The main function of PTEN is to negatively regulate PI3K-AKT signaling pathway, which can activate the AKT and its downstream gene p-Akt (S473), p-Akt (T308), Akt, p-mTOR, mTOR, p-4E-BP1, 4E-BP1, p-S6K, and S6K through phosphorylation to promote cell proliferation, migration, and anti-apoptosis. Therefore, we used Western blotting to determine the protein expression of p-Akt (S473), p-Akt (T308), Akt, p-mTOR, mTOR, p-4E-BP1, 4E-BP1, p-S6K, and S6K in cells after transfection with mimic *miR-500a* or inhibitor *miR-500a*. Total proteins from the cells were extracted by ice-cold radioimmunoprecipitation assay (RIPA) lysis buffer supplemented with 1 mM proteinase inhibitor PMSF (Sigma, St. Louis, MO, U.S.A.). The protein concentration was quantitated with a BCA assay kit (Beyotime, Shanghai, China). Equal amounts of protein were separated by SDS/PAGE (10% gel), transferred on to PVDF (Millipore, Bedford, MA, U.S.A.) membrane, and then blocked with 5% non-fat milk in TBS. The membranes were incubated with primary antibodies, mouse anti-human monoclonal PTEN, Akt, mTOR, 4E-BP1, and S6K antibody (Santa Cruz Biotechnology, CA, U.S.A.) and mouse anti-human monoclonal β-actin antibody (Santa Cruz Biotechnology, CA, U.S.A.), at 4°C overnight. The membranes were washed and subsequently probed with secondary antibody, goat anti-rabbit IgG conjugated to horseradish peroxidase (Santa Cruz Biotechnology, Santa Cruz, CA, U.S.A.) at a 1/4000 dilution for 1 h at room temperature. Proteins were visualized with chemiluminescent detection system (ECL; Beyotime). Glyceraldehyde-3-phosphate dehydrogenase (GAPDH) was used as internal control.

### Cell viability assay

Cells were seeded in the 96-well plate for 24 h after transfected at a density of 1500 cells/well. The cell viability assay was performed using Cell Counting Kit-8 (CCK8; Dojindo) according to the manufacturer’s protocol every 2 days. The absorbance at 450 nm was measured. Experiments were performed thrice.

### Cell invasion assay

Cell invasion assay was performed using 24-well transwell chambers containing 8-mm pore diameter polycarbonate membrane (Corning, New York, NY, U.S.A.). Two hundred microliters of cell suspension containing 4 × 10^4^ cells were added into the upper chamber, and 500 μl culture medium containing 10% (v/v) FBS was added into the lower chamber. After incubation at 37°C under 5% (v/v) CO_2_ for 24 h, the non-filtered cells were gently removed with a cotton swab, and the migrated cells were fixed with 100% methanol, stained with 0.5% Crystal Violet and washed with PBS (Gibco). The invaded cell number was counted under the microscope.

### Luciferase activity assays

Wild-type and mutant 3′-UTR of PTEN sequences were cloned into the psi-mediated instrumental response (pMIR) luciferase reporter vector (Thermo Fisher, U.S.A.). For the luciferase assays, 100 ng pMIR luciferase reporter vector was co-transfected in cells with 100 nM *miR-500a* mimics or control regent, together with 20 ng pMIR-REPORT β-gal Control Plasmid (Thermo Fisher, U.S.A.) as an internal normalized control. Cells were harvested 48 h after transfection and the luciferase activities were assayed according to the manufacturer’s protocol. Transfections were performed in duplicate and repeated three times.

### Clone formation

Cell suspension (5 × 10^6^ cells/ml) of SMMC-7721 was seeded into two 60-mm Petri dishes with 2 × 10^2^ cells in each dish. The cells were dispersed evenly by slightly shaking the Petri dishes and were then incubated at 37°C with 5% CO_2_ for 21 days until the visible clones appeared. The medium was discarded and the cells were carefully washed with PBS twice. After being fixed with methanol for 15 min, the cells were stained with Giemsa’s solution for 15 min before washing with tap water and air drying. The clones with more than 50 cells were counted with an ordinary optical microscope and the clone formation rate was calculated with the following formula: plate clone formation efficiency = (number of clones/number of cells inoculated) × 100%. All the experiments were repeated three times and the average values were reported.

### Statistical analysis

Statistical analyses were performed using SPSS (SPSS Inc., Chicago, IL, U.S.A.). All data were expressed as mean ± S.D. Nonparametric test was performed to determine significant differences. A *P*<0.05 was considered statistically significant.

## Results

### *MiR-500a* was up-regulated in hepatocarcinoma metastasis patients

A previous study showed that *miR-500* was abundantly expressed in several human liver cancer cell lines and 45% of human HCC tissue [9]. To explore the influence of *miR-500a* on hepatocarcinoma, serum was obtained from hepatocarcinoma patients and the normal people, and the relative RNA level of *miR-500a* in them was determined and compared. Our study showed that the expression of serum *miR-500* in hepatocarcinoma patients was significantly higher than the normal people (Figure 1A). To study the relationship between *miR-500a* and tumor metastasis, we studied the level of *miR-500a* in serum from metastatic and non-metastatic hepatocarcinoma patients. Results showed that the expression of serum *miR-500a* was significantly increased in metastatic hepatocarcinoma patients than non-metastatic ones (Figure 1B). Moreover, the expression of *miR-500a* in hepatocarcinoma tissue was dramatically higher than the adjacent tissues in metastatic and non-metastatic patients (Figure 1C). These indicated that *miR-500a* has the potential to be used as a biomarker for hepatocarcinoma detection.

**Figure 1:** Expression of *miR-500a* was increased in serum and tissues of patients with hepatocarcinoma (**A**) Serum *miR-500a* expression was significantly increased in hepatocarcinoma patients compared with the normal people. (**B**) Serum *miR-500a* expression was significantly increased in metastatic hepatocarcinoma patients than non-metastatic ones. (**C**) Expression of *miR-500a* was significantly increased in tumor tissues compared with the adjacent tissue in metastatic and non-metastatic hepatocarcinoma patients. **P<0.01, compared with the non-metastatic group, the relative *miR-500a* expression in metastatic group had a significant difference.

### Overexpression of *miR-500a* promoted the proliferation and invasion of hepatocarcinoma

To investigate the effect of *miR-500a* in hepatocarcinoma cell proliferation, SMMC-7721 cells were treated with mimic *miR-500a* and inhibitor *miR-500a* for 2, 4, and 6 days. qRT-PCR was used to verify the transfection effect. Results showed that the expression level of *miR-500a* increased significantly after transfection with mimic *miR-500a* (Figure 2A) and decreased observably after transfection with inhibitor *miR-500a* (Figure 2C). Cell proliferation assay revealed that relative SMMC-7721 cell number increased significantly after transfection with mimic *miR-500a* for 4 and 6 days (Figure 2B), and decreased dramatically after transfection with inhibitor *miR-500a* for 2, 4, and 6 days (Figure 2D). Moreover, a transwell assay showed that overexpression of *miR-500a* significantly promoted the invasion of SMMC-7721 cells compared with the cells transfected with mimic NC (Figure 2E,F), while knockdown of *miR-500a* inhibited the invasion of cells compared with the cells transfected with inhibitor NC (Figure 2G,H).

**Figure 2:** *MiR-500a* regulated the proliferation in SMMC-7721 cells (**A,B**) Transfection of mimic *miR-500a* increased *miR-500a* level, while inhibitor *miR-500a* decreased the level. RNA expression was measured by real-time PCR. *P<0.05 and **P<0.01, compared with mimic *miR-500a* group, the relative cell number in mimic NC group had a significant difference. (**C,D**) Transfection with mimic *miR-500a* accelerated SMMC-7721 cell proliferation, while inhibitor *miR-500* inhibited cell proliferation. Cell proliferation was measured by CCK8 kit in after transfection with mimic or inhibitor *miR-500* for 0, 2, 4, and 6 days. *P<0.05 and **P<0.01, compared with inhibitor *miR-500a* group, the relative cell number in inhibitor NC group had a significant difference. (**E,F**) Cell invasion ability was increased when transfected with mimic *miR-500a* in SMMC-7721 cells. (**G,H**) Cell invasion ability was decreased when transfected with inhibitor *miR-500a* in SMMC-7721 cells. Cell invasion abilities were measured by a transwell assay method after transfection for 48 h. **P<0.01, compared with the NC group, the relative or average cell number in mimic *miR-500a* or inhibitor *miR-500a* group had significant difference.

### Overexpression of *miR-500a* increased the cloning of hepatocarcinoma cells

As the above results showed, we obtained that the overexpression of *miR-500a* promoted the proliferation capacity of hepatocarcinoma cells. To further explore the influence, we cloned SMMC-7721 cells after transfection with mimic *miR-500a* and inhibitor *miR-500a*. Results showed that the clone number of SMMC-7721 cells was significantly increased after transfection with mimic *miR-500a* compared with the mimic NC group and decreased after transfection with inhibitor *miR-500a* compared with the inhibitor NC group (Figure 3A–D).

**Figure 3:** *MiR-500a* regulated clone formation in SMMC-7721 cells (**A**) Clone formation was increased when transfected with mimic *miR-500a* in SMMC-7721 cells. (**B**) The column diagram about the average clone number in mimic NC and mimic *miR-500a* group. **P<0.01, compared with the mimic NC group, the average clone number of SMMC-7721 cells in mimic *miR-500a* had a significant difference. (**C**) Clone formation was decreased when transfected with inhibitor miR-500a in SMMC-7721 cells. (**D**) The column diagram about the average clone number in inhibitor NC and inhibitor *miR-500a* group. *P<0.05, compared with the inhibitor NC group, the average clone number of SMMC-7721 cells in inhibitor *miR-500a* had a significant difference.

### PTEN is a direct target of *miR-500a* in hepatocarcinoma

By target gene prediction analysis, we found that there had been binding sites between PTEN and miRNA. To explore whether PTEN was a direct target for *miR-500a*, we constructed the 3′-UTR reporter plasmids coupled with full length of PTEN 3′-UTR with wild-type (wt) or mutant (mut) *miR-500*-binding sites (Figure 4A). Luciferase assay showed that *miR-500a* could repress the expression of reporter gene containing wt 3′-UTR but not that containing mut 3′-UTR (Figure 4B). Then, we determined the protein expression values of PTEN, p-Akt (S473), p-Akt (T308), Akt, p-mTOR, mTOR, p-4E-BP1, 4E-BP1, p-S6K, and S6K in SMMC-7721 cells after transfection with mimic NC, mimic *miR-500a*, inhibitor NC, and inhibitor *miR-500a*. Results showed that the protein expression of PTEN was significantly decreased after transfection with mimic miR-500a, while the expression was increased observably after transfection with inhibitor miR-500a (Figure 4C,D). The protein expression values of p-Akt (S473)/Akt, p-mTOR/mTOR, and p-4E-BP1/4E-BP1 were increased observably after transfection with mimic *miR-500a*, while the expression was significantly decreased after transfection with inhibitor *miR-500a* (Figure 4E,G,H). The protein expression of p-Akt (T308)/Akt and p-S6K/S6K were decreased observably after transfection with inhibitor *miR-500a*, while transfection of mimic *miR-500a* had no influence on the expression values (Figure 4F,I).

**Figure 4:** PTEN was the target gene of *miR-500a* (**A**) Diagram of the *miR-500a* putative binding sites and corresponding mutant sites in the 3′-UTR of PTEN. (**B**) Effects of *miR-500a* on the expression of PTEN 3′-UTR-containing reporter genes. (**C**) The protein expression of PTEN, p-Akt (S473), p-Akt (T308), Akt, p-mTOR, mTOR, p-4E-BP1, 4E-BP1, p-S6K, and S6K in SMMC-7721 cells after transfection with mimic *miR-500a* or inhibitor *miR-500a*. (**D**–**I**) The relative optical density of PTEN, p-Akt (S473)/Akt, p-Akt (T308)/Akt, p-mTOR/mTOR, p-4E-BP1/4E-BP1, and p-S6K/S6K in SMMC-7721 cells after transfection with mimic *miR-500a* or inhibitor miR-500a. *P<0.05 and **P<0.01, compared with the NC group, the relative optical density in mimic *miR-500a* or inhibitor *miR-500a* group had a significant difference.

## Discussion

Hepatocarcinoma is a common visceral malignancy and amongst the leading causes of cancer deaths worldwide. It typically arises in a setting of chronic hepatitis or cirrhosis, with infection by hepatitis B and C viruses and chronic exposure to aflatoxin B together responsible for ~80% of all hepatocarcinoma cases in humans [10]. miRNAs are a class of small noncoding RNAs that control gene expression by targetting mRNAs and triggering either translation repression or RNA degradation [11]. They have rapidly emerged as modulators of gene expression in cancer in which they may have great diagnostic and therapeutic importance [12]. *MiR-500a* is a key player in breast cancer survival and the expression of *miR-500a* is increased in highly tumorigenic derivative of MDA-MB-231 cell line compared with its low tumorigenic parental cell line [13]. Moreover, median levels of *miR-500a* were higher in HCC patients than in healthy controls [14].

Our study showed that the pre-miRNA level of serum *miR-500a* in hepatocarcinoma patients was significantly higher than the normal. The expression of serum *miR-500a* was significantly increased in metastatic hepatocarcinoma patients than non-metastatic ones. The level of *miR-500a* in hepatocarcinoma tumor tissues was dramatically increased compared with the adjacent tissues. It indicated that *miR-500a* was up-regulated in patients with hepatocarcinoma, which manifested that the expression of *miR-500a* was closely related with hepatocarcinoma. *MiR-500a-3p* was found to play a role in breast cancer proliferation as well as doxorubicin-induced cardiotoxicity [15]. To further explore the role of *miR-500a* on hepatocarcinoma, we transfected hepatocarcinoma cell lines SMMC-7721 with mimic *miR-500a* or inhibitor *miR-500a*, and then determined the proliferation, invasion, and cloning capacity of SMMC-7721 cells. Results showed that overexpression of *miR-500a* increased the proliferation, invasion, and cloning capacity of SMMC-7721 cells, while knockdown of *miR-500a* decreased the capacity. It further verified the role of *miR-500a* on hepatocarcinoma.

PTEN can be used clinically to suppress tumor and inhibit the activation of PI3K/AKT signaling pathway [16]. The loss of PTEN can result in the activation of AKT kinases, which play key roles in cell growth, proliferation, and invasion [17]. Here, we identified PTEN as a direct and functional target of *miR-500a*. Study showed *miR-500a* overexpression inhibited the expression of PTEN. The protein expression values of PTEN, p-Akt (S473), p-Akt (T308), Akt, p-mTOR, mTOR, p-4E-BP1, 4E-BP1, p-S6K, and S6K in SMMC-7721 cells after transfection with mimic NC, mimic *miR-500a*, inhibitor NC, and inhibitor *miR-500a* were determined by Western blotting. Results showed overexpression of *miR-500a* decreased the expression of PTEN, while increased the expression of Akt, mTOR, and 4E-BP1. As previous studies reported PI3K/AKT/mTOR pathway was regulated by miRNA and PI3K/Akt signal transduction cascade was reported to have roles in oncogenic transformation [18,19]. The PI3K/AKT signaling pathway prevents apoptosis of mature hepatocytes and HCC cells [20]. mTOR is a large protein kinase and the target of rapamycin, an immunosuppressant that also blocks vessel restenosis and has potential anticancer applications [21]. It controls multiple cellular functions in response to amino acids and growth factors, in part by regulating p70S6k and 4E-BP1 [22]. In this study, overexpression of *miR-500a* increased the phosphorylation of both mTOR and 4E-BP1. All these indicated that the up-regulated *miR-500a* decreased the expression of PTEN, and the loss of PTEN activated AKT/mTOR signaling pathway which promoted the metastasis of hepatocarcinoma.

In summary, our results showed that *miR-500a* could promote hepatocarcinoma proliferation, invasion, and metastasis by regulating PTEN via activating AKT/mTOR signaling pathway.

## Abbreviations

HCC: hepatocellular carcinoma
GAPDH: Glyceraldehyde-3-phosphate dehydrogenase
pMIR: psi-mediated instrumental response
pre-miRNA: precursor miRNA
PTEN: phosphatase and tensin homologue
qRT-PCR: quantitative reverse transcription-PCR
RIPA: radioimmunoprecipitation assay
